The article "Obesity and Frailty Syndrome in the Elderly: Prospective Study in Primary Care" was retracted in 2024. Reasons: lack of ethics approval or compliance; concerns about the welfare of human subjects.

# Obesity and Frailty Syndrome in the Elderly: Prospective Study in Primary Care

**DOI:** 10.3390/medicines9070038

**Published:** 2022-06-24

**Authors:** Abrar-Ahmad Zulfiqar, Perla Habchi, Ibrahima Amadou Dembele

**Affiliations:** 1 Service de Médecine Interne, Diabète et Maladies Métaboliques de la Clinique Médicale B, Hôpitaux Universitaires de Strasbourg et Equipe EA 3072 “Mitochondrie, Stress Oxydant et Protection Musculaire”, Faculté de Médecine-Université de Strasbourg, 67000 Strasbourg, France; ibrahimaadembele@gmail.com; 2 Anesthesiology Consultant, Aman Hospital, F Ring Rd, Zone 47, Building 412, Doha P.O. Box 8199, Qatar; p.habchi@amanhospital.org

**Keywords:** obesity, frailty syndrome, Fried’s scale, sZFS, sarcopenic obesity, primary care

## Abstract

*Background:* Obesity is a chronic pathology that affects people of all ages, from infants to the elderly, residing in both developed and developing countries. *Objective:* Our aim is to study the link between obesity and frailty in the elderly. *Method:* A prospective study was carried out in 12 General Medicine practices in Champagne-Ardenne, in the Departments of Marne and the Ardennes, France, for a period of 12 months (from 2 May 2019 through 30 April 2020). All patients included were aged 65 or older, in consultation with a general practitioner, and had an ADL (Activity of Daily Living) greater than or equal to 4. Frailty was measured using the Fried scale and the simplified ZULFIQAR frailty scale. *Results:* 268 patients aged 65 and over were included, with an average age of 77.5 years. A total of 100 were obese according to BMI. The mean Fried (/5) in the series was 1.57, and the mean sZFS (/5) was 0.91. Our study shows that obesity is not significantly correlated with frailty according to the FRIED sarcopenic scale, but is significantly correlated with frailty according to the sZFS scale. *Conclusions:* The link between obesity and frailty remains much debated, with the underlying emergence of sarcopenic obesity equally prevalent among the elderly. This is a preliminary study that should be followed by large-scale outpatient studies to better clarify the links between sarcopenia and obesity.

## 1. Introduction

The international World Health Organization (WHO) Consultation on Obesity of 1997 defined obesity as “an abnormal or excessive accumulation of fat in adipose tissue that could cause health problems” [1]. Obesity is a chronic pathology that affects people of all ages, from infants to the elderly, residing in both developed and developing countries. In the United States, the prevalence of obesity alone is over 40%—almost equal to the prevalence of overweightness and obesity combined in France. One study recently published in the *New England Journal of Medicine* predicts that the prevalence of obesity will reach 50%, and severe obesity 25%, by the end of the decade [2]. In France, the ESTEBAN study (the Health Study on the Environment, Biomonitoring, Physical Activity and Nutrition) was published in 2017 [3]. It looked at subjects between the ages of 6 and 74, studying the dietary habits, physical activity, risk factors and chronic illnesses of the French population. Piloted by the French Public Health Agency, it was part of the French National Nutrition and Health Program. Based on a sample of 2503 adults, the study found an average BMI of 25.8 among men, and 25.7 among women–both classified as “overweight.” One out of every two subjects (49%) was classified as either overweight or obese, with a significantly higher portion of those being male (53.0%) than female (44.2%). The prevalence of obesity was 17.2%, with no significant difference between genders, which is higher than its prevalence worldwide (13%). This study also revealed an increase in the prevalence of overweightness and obesity as age increases, regardless of gender. The prevalence of obesity was above 20% among subjects of any gender over the age of 55. Very few studies have been carried out on obesity in the very elderly, an age category also subject to concerns of frailty. The main objective of our study was to study the relationship between obesity and frailty in an outpatient population based on the Fried scale [4] and the simplified ZULFIQAR frailty scale, known as sZFS [5,6]. This simplified scale was derived from the Zulfiqar Frailty Scale (sZFS) and included five items (one item regarding social interactions—the question, “Does the patient benefit from home care?”—was removed). The sZFS was validated in two studies which were published [5,6].

The article "Obesity and Frailty Syndrome in the Elderly: Prospective Study in Primary Care" was retracted in 2024. Reasons: lack of ethics approval or compliance; concerns about the welfare of human subjects.

## 2. Methodology

### 2.1. Study Type 

To answer our research questions, a prospective and observational study was designed and carried out in 12 General Medicine practices in Champagne-Ardenne, in the Departments of Marne (51) and the Ardennes (08), for a period of 12 months (from 2 May 2019 through 30 April 2020).

### 2.2. Study Population

Our study population was made up of patients aged 65 or older who were monitored by a general practitioner and had an ADL (Activities of Daily Living) score of 4/6 or higher. Patients who did not provide their verbal consent during the introductory phase of the study, were under 65 years of age, had an ADL score of less than 4/6, or lived in nursing homes were excluded from the study. 

### 2.3. Study Parameters 

#### 2.3.1. Population Characteristics

The data collected were: gender, age, the Activity (Katz Index of ADL) and Instrumental (Lawton Index of IADL) of daily living score, the medical comorbidities needed to calculate the Charlson comorbidity index, treatment background, weight, height, and BMI calculation. The number and nature of any regular treatments were also recorded.

#### 2.3.2. Frailty Screening with the “Simplified Zulfiqar Frailty Scale” (sZFS) Tool

The score was calculated by way of five indicators that measured the main functions of an elderly person in terms of their geriatric relevance as defined by the scientific literature. A point was assigned for each positive indicator (maximum score = 5) [5,6].

- Nutritional status: weight loss of 5% or more during the previous 6 months
- Physical capabilities, balance/falls: one-legged stance test.
- Social isolation: does the patient live at home alone?
- Cognitive functions: does the patient complain of memory loss?
- Polymedicine: the patient has been taking 5 or more types of medications for at least 6 months.

#### 2.3.3. Frailty Screening with the Fried Scale

Fried’s scale [4] defines frailty on the basis of 5 criteria: fatigue, involuntary weight loss, reduced physical activity, slower walking speed, and decreased muscle strength. A point is assigned for each criterion, with patients considered “robust” or “non-frail” when none of the criteria are met, “pre-frail” when 1 or 2 of the criteria are met, and “frail” when 3 or more of the criteria are met.

### 2.4. Statistical Analysis

Statistical analysis was performed using R 3.6.1 software. The qualitative variables were translated into numerical values and percentages by response modality. Quantitative variables were expressed as means and standard deviations. Bivariate analyses were performed to compare people with diabetes to people without diabetes. Student tests were carried out to compare the means, or Wilcoxon tests when the conditions for applying the parametric tests were not met. The proportions were compared using Chi-square tests, or Fisher tests when there were insufficient data. All tests were bilateral and were considered significant if the *p*-value was less than 0.05.

### 2.5. Administrative Elements

Informed consent was obtained from all patients included in this study. In terms of regulatory compliance, the study was registered with the CNIL (National Commission for Computing and Liberties) according to the MR-004 reference methodology, and in the Heath Data Hub directory. The research protocol was reviewed and approved by the National Commission of Information and Freedom and by the Internal Department Ethics Committee (No. 20-06-19).

## 3. Results

### 3.1. Description of Population

Data were collected from 268 patients aged 65 and over. In this population, the average age is 77.5, with a male-to-female ratio of 1.144. There were no refusals noted. The characteristics of the population included are detailed in Table 1. 

The article "Obesity and Frailty Syndrome in the Elderly: Prospective Study in Primary Care" was retracted in 2024. Reasons: lack of ethics approval or compliance; concerns about the welfare of human subjects.

### 3.2. Comparison of Obese and Non-Obese Elderly Patients

Table 2 shows the results of the comparison between the obese elderly and non-obese elderly outpatient populations.

### 3.3. Primary Criteria of Interest

This study focused on obesity, as defined by BMI, shown in Table 3. This table shows that obesity is not significantly correlated with frailty according to the FRIED sarcopenic scale, but is significantly correlated with frailty according to the sZFS scale (Table 3).

## 4. Discussion 

Literature has established that obesity is associated with increased risk of developing cardiovascular disease, hypertension, coronary artery disease, heart failure, stroke, and death [7,8,9,10,11,12]. It represents an epidemic with far-reaching consequences on health and morbidity. In the review of scientific literature, the links between obesity and frailty syndrome in the elderly are beginning to be discussed, with contradictory results. Tamura et al. analyzed the most prominent studies related to nutritional pathologies and frailty [13]. Schaap et al. showed an increase in functional decline and a decrease in physical strength in elderly subjects with a BMI over 30 [14]. In contrast, García-Esquinas et al. seemed to find a reduced risk of frailty with obesity in multivariate analysis [15]. Nam et al. saw a protective effect against cognitive impairment when BMI was high, and a higher incidence when BMI was low [16]. In a Japanese study by Watanabe et al., a U-shaped relationship was found between BMI and frailty–the lowest risk being observed with a BMI between 21.4 and 25.7 kg/m^2^ [17]. Xu et al. found similar results in a Chinese study of 656 elderly subjects: malnutrition, a high waist circumference (H > 102/ F > 88), a high percentage of fat and a low percentage of muscle mass were significantly associated with an increased risk of frailty, assessed by the Clinical Frailty Scale (CFS) [18].

Few articles or scientific works have been produced in the field of frailty obesity with the use of frailty scales. Ting MJM et al. conducted a prospective cohort study of 4219 older men to investigate if diabetes and obesity are associated with frailty independently; frailty syndrome was measured by the FRAIL scale. Diabetes and obesity were found to be modifiable risk factors which independently carry equal risk for the development of frailty in older men [19]. 

Bhardwaj PV et al. found no relationship between BMI and frailty among 769 hospitalized older adults, with frailty syndrome measured by the Reported Edmonton Frailty Scale (REFS) [20].

The article "Obesity and Frailty Syndrome in the Elderly: Prospective Study in Primary Care" was retracted in 2024. Reasons: lack of ethics approval or compliance; concerns about the welfare of human subjects.

Another study using the Clinical Frailty Scale (CFS), aimed at investigating the association between body composition and frailty in elderly inpatients, showed that the body composition of frail elderly inpatients was characterized by low skeletal muscle mass, underweight and high body fat mass, and high waist circumference compared with non-frail inpatients [18].

Ahmed AM conducted a study with the aim of describing the prevalence and predictors of frailty among Saudi patients referred for cardiac stress testing with nuclear imaging. The Fried Clinical Frailty Scale was used to assess frailty. In a fully adjusted logistic regression model, women, hypertension, and obesity (BMI ≥ 30 kg/m^2^) were independent predictors of elderly frail patients [21]. 

Our study, carried out on an outpatient basis, shows a link between obesity and frailty as measured by the simplified ZULFIQAR scale, but not as measured by Fried’s sarcopenic scale. This can be explained by the small sample size; the monocentric nature of the study, which was carried out in a single general practice; but also by the fact that the elderly subjects included are outpatients. This is the first prospective study conducted in primary care, evaluating a link between obesity and frailty syndrome in elderly outpatients in France.

A new concept has recently been introduced to the world of geriatric medicine: Sarcopenic Obesity [22]. It is defined by the concomitant presence of obesity and sarcopenia [22]. If, by consensus, sarcopenia is established before a loss of muscle mass and muscle weakness, obesity can be established either by a BMI > 30, or by a waist circumference above the limit. Hirani et al. showed a higher prevalence of frailty and decreased autonomy associated with sarcopenic obesity [22]. Moreover, sarcopenic obesity seems to be more frequently found in diabetic patients. These patients would, according to Kim et al., show a significantly lower percentage of muscle mass as well as a BMI and body fat percentage greater than or equal to non-diabetics [23]. 

Sarcopenic obesity is strongly associated with frailty, cardiometabolic dysfunction, physical disability, and mortality [24]. This concept of sarcopenic obesity has emerged and is considered a public health risk in older adults [25,26,27]. Sarcopenia and obesity are both considered multifactorial syndromes sharing various overlapping causes and feedback mechanisms. However, different studies have presented confusing views on the pathogenic relationship between sarcopenia and obesity, with no clear answer [18,25]. Inflammation and insulin resistance both play important roles in sarcopenia and obesity, but the origins of local inflammation and insulin resistance, and how they cause systemic inflammation, systemic insulin resistance, and changes in body composition, had remained unclear [27]. Numerous molecules (TNF-α, IL-6, IL-1, adiponectin, leptin, muscle somatostatin, sex hormones (testosterone and estrogen), growth hormone, insulin and glucocorticoid, and irisin) have been implicated in the pathogenesis of sarcopenic obesity [28,29]. Sarcopenic obesity is the concurrence of muscle loss and excessive body fat accrual [27,28]. Korea’s recommended sarcopenic obesity diagnostic criteria are defined as subjects fulfilling both the criteria for obesity (men with body fat ≥ 27%, and women with body fat ≥ 38%) and the European Working Group on Sarcopenia in Older People 2 (EWGSOP2) criteria for sarcopenia [30]. The core mechanism of sarcopenic obesity is the vicious circle between myocytes and adipocytes [31]. In a cross-sectional study involving data from the Korean Frailty and Aging Cohort Study, central obesity was associated with a low prevalence of sarcopenia in women only. This was the first large cross-sectional cohort study to investigate the association between obesity and the component parameters of sarcopenia [32].

The article "Obesity and Frailty Syndrome in the Elderly: Prospective Study in Primary Care" was retracted in 2024. Reasons: lack of ethics approval or compliance; concerns about the welfare of human subjects.

The main limitation lies in the monocentric nature of the study, with a small sample size. It will be important to replicate this study in additional general medical practices. Moreover, the association between body fat indices measured using dual-energy DXA and sarcopenia was not included in our study. In follow-up research, sarcopenia should be studied via dual-energy X-ray absorptiometry (DXA) and bioelectrical impedance analysis, not just weight and BMI.

## 5. Conclusions

The links between obesity and frailty remain much debated, with the underlying emergence of sarcopenic obesity equally prevalent among the elderly. This is a preliminary study that should be followed by large-scale outpatient studies to better clarify the links between frailty syndrome and obesity.

## Figures and Tables

**Table 1:** Description of the sample population.

		N = 268
Sex, n (%)	Female	125 (46.6)
	Male	143 (53.4)
Age, m (sd)		77.5 (7.8)
Place of residence, n (%)	Rural	163 (60.8)
	Urban	105 (39.2)
Marital status, n (%)	Married	166 (61.9)
	Divorced/Single	16 (6.0)
	Widowed	86 (32.1)
Diabetes, n (%)		129 (48.1)
Type of diabetes, n (%)	I	4 (3.1)
	II	125 (96.8)
Duration, in years, m (sd)		15.2 (9.3)
HbA1c, m (sd)		7.32 (1.25)
Renal disease, n (%)		81 (62.8)
Eye disease, n (%)		19 (14.7)
Heart disease, n (%)		37 (28.7)
Diabetic foot, n (%)		12 (9.3)
Neuropathy, n (%)		22 (17.0)
Obliterating arteriopathy, n (%)		24 (18.6)
Other, n (%)		1 (0.8)
Weight, in kilos, m (sd)		79.9 (16.5)
Height, in centimeters, m (sd)		165.7 (8.9)
BMI in kg/m², m (sd)		29.1 (5.3)
Nutritional status, according to BMI, n (%)	Malnourished	8 (3.0)
	Normal	52 (19.4)
	Overweight	108 (40.3)
	Obese	100 (37.3)
Smoking status, n (%)	Non-smoker	140 (52.2)
	Former smoker	93 (34.7)
	Smoker	35 (13.1)
ADL, out of 6, m (sd)		5.60 (0.90)
IADL, out of 4, m (sd)		0.72 (1.08)
Charlson, out of 24, m (sd)		2.43 (1.92)
Fried, out of 5, m (sd)		1.57 (1.12)
Weight, n (%)		17 (6.3)
Fatigue, n (%)		7 (2.6)
Mobility, n (%)		176 (65.7)
Activity, n (%)		149 (55.6)
Strength, n (%)		72 (26.9)
sZFS, out of 5, m (sd)		0.91 (0.88)
Weight, n (%)		16 (6.0)
Monopedal balance, n (%)		128 (47.8)
Isolation, n (%)		63 (23.5)
Memory, n (%)		35 (13.1)
Polypharmacy, n (%)		3 (1.1)
Number of treatments, m (sd)		7.59 (3.84)
Antihypertensive drugs, n (%)		225 (83.9)
Antiplatelet agents, n (%)		117 (43.7)
Anticoagulants, n (%)		45 (16.8)
Oral antidiabetics, n (%)		106 (39.6)
Insulin, n (%)		40 (14.9)

BMI: Body Mass Index; ADL: Activity of Daily Living; IADL: Instrumental of Activity of Daily Living; sZFS: simplified Zulfiqar Frailty Scale.

The article "Obesity and Frailty Syndrome in the Elderly: Prospective Study in Primary Care" was retracted in 2024. Reasons: lack of ethics approval or compliance; concerns about the welfare of human subjects.

**Table 2:** Comparing the characteristics of obese and non-obese patients.

Data Collected		Non Obese	Obese	*p*
n		168	100	
Sex (%)	Female	79 (47.0)	46 (46.0)	0.971
	Male	89 (53.0)	54 (54.0)	
Age (mean (SD))		78.93 (7.99)	74.99 (6.78)	<0.001
Location (%)	Rural	98 (58.3)	65 (65.0)	0.341
	Urban	70 (41.7)	35 (35.0)	
Marital status (%)	Divorced/Single	8 (4.8)	8 (8.0)	0.009
	Married	95 (56.5)	71 (71.0)	
	Widower	65 (38.7)	21 (21.0)	
Diabetes (%)	No	94 (56.0)	45 (45.0)	0.108
	Yes	74 (44.0)	55 (55.0)	
Type of diabetes (%)	I	2 (1.2)	2 (2.0)	1.000
	II	72 (42.9)	53 (53.0)	
Duration of diabetes (mean (SD))		14.51 (7.97)	16.11 (10.90)	0.339
HbA1c (mean (SD))		7.19 (1.12)	7.50 (1.40)	0.174
Renal disease (%)	No	23 (13.7)	25 (25.0)	0.137
	Yes	51 (30.4)	30 (30.0)	
Retinopathy (%)	No	68 (40.5)	42 (42.0)	0.027
	Yes	6 (3.6)	13 (13.0)	
Heart disease (%)	No	52 (31.0)	40 (40.0)	0.914
	Yes	22 (13.1)	15 (15.0)	
Diabetic foot (%)	No	68 (40.5)	49 (49.0)	0.814
	Yes	6 (3.6)	6 (6.0)	
Neuropathy (%)	No	63 (37.5)	44 (44.0)	0.596
	Yes	11 (6.5)	11 (11.0)	
Obliterating arteritis (%)	No	66 (39.3)	39 (39.0)	0.016
	Yes	8 (4.8)	16 (16.0)	
Other (%)	No	74 (44.0)	54 (54.0)	0.426
	Yes	0 (0.0)	1 (1.0)	
Weight (mean (SD))		71.02 (10.79)	94.84 (13.35)	<0.001
Height (mean (SD))		166.04 (8.78)	165.17 (9.14)	0.443
BMI (mean (SD))		25.75 (2.60)	34.76 (3.77)	<0.001
Nutrition status (%)	Malnutrition	8 (4.8)		
	Normal	52 (31.0)		
	Overweight	108 (64.3)		
Smoker (%)	Former smoker	51 (30.4)	42 (42.0)	0.035
	Smoker	19 (11.3)	16 (16.0)	
	None smoker	98 (58.3)	42 (42.0)	
ADL /6 (mean (SD))		5.56 (1.01)	5.67 (0.69)	0.301
IADL/4 (mean (SD))		0.73 (1.11)	0.70 (1.02)	0.822
CHARLSON/24 (mean (SD))		2.29 (1.98)	2.65 (1.80)	0.139
FRIED/5 (mean (SD))		1.57 (1.15)	1.57 (1.08)	0.975
FRIED weight (%)	0	158 (94.0)	93 (93.0)	0.935
	1	10 (6.0)	7 (7.0)	
FRIED fatigue (%)	0	165 (98.2)	96 (96.0)	0.430
	1	3 (1.8)	4 (4.0)	
FRIED walk (%)	0	55 (32.7)	37 (37.0)	0.563
	1	113 (67.3)	63 (63.0)	
FRIED activity (%)	0	78 (46.4)	41 (41.0)	0.461
	1	90 (53.6)	59 (59.0)	
FRIED strength (%)	0	120 (71.4)	76 (76.0)	0.500
	1	48 (28.6)	24 (24.0)	
sZFS/5 (mean (SD))		0.98 (0.95)	0.80 (0.75)	0.103
sZFS weight (%)	0	158 (94)	94 (94)	1.000
	1	10 (6)	6 (6)	
sZFS monopodal balance (%)	0	87 (51.8)	53 (53)	0.947
	1	81 (48.2)	47 (47)	
sZFS isolation (%)	0	124 (73.8)	81 (81)	0.233
	1	44 (26.2)	19 (19)	
sZFS mémory (%)	0	140 (83.3)	93 (93)	0.037
	1	28 (16.7)	7 (7)	
sZFS polymedication (%)	0	166 (98.8)	99 (99)	1.000
	1	2 (1.2)	1 (1)	
Number of treatments (mean (SD))		6.81 (3.69)	8.91 (3.75)	<0.001
Number of antihypertensive treatments (mean (SD))		1.83 (1.30)	2.37 (1.31)	0.001
Antiplatelet agents (%)	No	99 (58.9)	52 (52.0)	0.328
	Yes	69 (41.1)	48 (48.0)	
Anticoagulants (%)	No	145 (86.3)	78 (78.0)	0.112
	Yes	23 (13.7)	22 (22.0)	
Oral antidiabetic treatment (%)	No	8 (4.8)	5 (5.0)	1.000
	Yes	61 (36.3)	45 (45.0)	
Number of Oral antidiabetic treatment (mean (SD))		1.74 (0.81)	2.09 (0.90)	0.038
Insulin (%)	No	48 (28.6)	31 (31.0)	0.506
	Yes	21 (12.5)	19 (19.0)	

BMI: Body Mass Index; ADL: Activity of Daily Living; IADL: Instrumental of Activity of Daily Living; sZFS: simplified Zulfiqar Frailty Scale.

The article "Obesity and Frailty Syndrome in the Elderly: Prospective Study in Primary Care" was retracted in 2024. Reasons: lack of ethics approval or compliance; concerns about the welfare of human subjects.

**Table 3:** Study correlation between obesity and frailty syndrome.

Weight	Value	Fried (Mean (SD))	sZFS (Mean (SD))
**Malnourished**	N = 8	1.25 (1.28)	0.25 (0.46)
**Normal**	N = 52	1.79 (1.07)	1.17 (0.98)
**Overweight**	N = 108	1.48 (1.17)	0.94 (0.93)
**Obese**	N = 100	1.57 (1.07)	0.80 (0.75)
		*p* = 0.350	*p* = 0.012

## Data Availability

The datasets used and/or analyzed during the current study are available from the corresponding author on reasonable request.

## References

[1] Organisation Mondiale de la Santé (2003). Obésité: Prévention et Prise en Charge de L’épidémie Mondiale. Rapport d’une Consultation de L’oms.

[2] Ward Z.J., Bleich S.N., Cradock A.L., Barrett J.L., Giles C.M., Flax C., Long M.W., Gortmaker S.L. (2019). Projected U.S. State-Level Prevalence of Adult Obesity and Severe Obesity. N. Engl. J. Med..

[3] Equipe de Surveillance et D’épidémiologie Nutritionnelle (Esen) (2017). Etude de Santé sur L’environnement, la Biosurveillance, L’activité Physique et la Nutrition (Esteban) 2014–2016.

The article "Obesity and Frailty Syndrome in the Elderly: Prospective Study in Primary Care" was retracted in 2024. Reasons: lack of ethics approval or compliance; concerns about the welfare of human subjects.

[4] Fried L.P., Tangen C.M., Walston J., Newman A.B., Hirsch C., Gottdiener J., Seeman T., Tracy R., Kop W.J., Burke G. (2001). Cardiovascular Health Study Collaborative Research Group. Frailty in older adults: Evidence for a phenotype. J. Gerontol. A Biol. Sci. Med. Sci..

[5] Zulfiqar A.A., Dembélé I. (2021). Zulfiqar Frailty Scale: Overview, Stakes, and Possibilities. Medicines.

[6] Zulfiqar A.A. (2021). Validation of a new frailty scale in primary care: The simplified Zulfiqar frailty scale. Transl. Med. Aging.

[7] Calle E.E., Thun M.J., Petrelli J.M., Rodriguez C., Heath C.W. (1999). Body-mass index and mortality in a prospective cohort of U.S. adults. N. Engl. J. Med..

[8] Diehr P., Bild D.E., Harris T.B., Duxbury A., Siscovick D., Rossi M. (1998). Body mass index and mortality in nonsmoking older adults: The cardiovascular health study. Am. J. Public Health.

[9] Peeters A., Barendregt J.J., Willekens F., Mackenbach J.P., Mamun A.A., Bonneux L., for NEDCOM, the Netherlands Epidemiology and Demography Compression of Morbidity Research Group (2003). Obesity in adulthood and its consequences for life expectancy: A life-table analysis. Ann. Intern. Med..

[10] Kenchaiah S., Evans J.C., Levy D., Wilson P.W., Benjamin E.J., Larson M.G., Kannel W.B., Vasan R.S. (2002). Obesity and the risk of heart failure. N. Engl. J. Med..

[11] Dunlap S.H., Sueta C.A., Tomasko L., Adams K.F. (1999). Association of body mass, gender and race with heart failure primarily due to hypertension. J. Am. Coll. Cardiol..

[12] Katzmarzyk P.T., Janssen I., Ardern C.I. (2003). Physical inactivity, excess adiposity and premature mortality. Obes. Rev..

[13] Tamura Y., Omura T., Toyoshima K., Araki A. (2020). Nutrition Management in Older Adults with Diabetes: A Review on the Importance of Shifting Prevention Strategies from Metabolic Syndrome to Frailty. Nutrients.

[14] Schaap L.A., Koster A., Visser M. (2013). Adiposity, muscle mass, and muscle strength in relation to functional decline in older persons. Epidemiol. Rev..

[15] García-Esquinas E., Graciani A., Guallar-Castillón P., López-García E., Rodríguez-Mañas L., Rodríguez-Artalejo F. (2015). Diabetes and risk of frailty and its potential mechanisms: A prospective cohort study of older adults. J. Am. Med. Dir. Assoc..

[16] Nam G.E., Park Y.G., Han K., Kim M.K., Koh E.S., Kim E.S., Lee M.-K., Kim B., Hong O.-K., Kwon H.-S. (2019). BMI, Weight Change, and Dementia Risk in Patients with New-Onset Type 2 Diabetes: A Nationwide Cohort Study. Diabetes Care.

[17] Watanabe D., Yoshida T., Watanabe Y., Yamada Y., Kimura M., Kyoto-Kameoka Study Group (2020). A U-Shaped Relationship between the Prevalence of Frailty and Body Mass Index in Community-Dwelling Japanese Older Adults: The Kyoto-Kameoka Study. J. Clin. Med..

The article "Obesity and Frailty Syndrome in the Elderly: Prospective Study in Primary Care" was retracted in 2024. Reasons: lack of ethics approval or compliance; concerns about the welfare of human subjects.

[18] Xu L., Zhang J., Shen S., Hong X., Zeng X., Yang Y., Liu Z., Chen L., Chen X. (2020). Association between Body Composition and Frailty in Elder Inpatients. Clin. Interv. Aging.

[19] Ting M.J.M., Hyde Z., Flicker L., Almeida O.P., Golledge J., Hankey G.J., Yeap B.B. (2022). Associations between diabetes, body mass index and frailty: The Western Australian Health in Men Study. Maturitas.

[20] Bhardwaj P.V., Rastegar V., Meka R., Sawalha K., Brennan M., Stefan M.S. (2021). The Association Between Body Mass Index, Frailty and Long-Term Clinical Outcomes in Hospitalized Older Adults. Am. J. Med. Sci..

[21] Ahmed A.M., Ahmed D., Alfaris M., Holmes A., Aljizeeri A., Al-Mallah M.H. (2020). Prevalence and predictors of frailty in a high income developing country: A cross-sectional study. Qatar Med. J..

[22] Hirani V., Naganathan V., Blyth F., Le Couteur D., Seibel M., Waite L.M., Handelsman D.J., Cumming R. (2017). Longitudinal associations between body composition, sarcopenic obesity and outcomes of frailty, disability, institutionalisation and mortality in community-dwelling older men: The Concord Health and Ageing in Men Project. Age Ageing.

[23] Kim T.N., Park M.S., Yang S.J., Yoo H.J., Kang H.J., Song W., Seo J.A., Kim S.G., Kim N.H., Baik S.H. (2010). Prevalence and determinant factors of sarcopenia in patients with type 2 diabetes: The Korean Sarcopenic Obesity Study (KSOS). Diabetes Care.

[24] Colleluori G., Villareal D.T. (2021). Aging, obesity, sarcopenia and the effect of diet and exercise intervention. Exp. Gerontol..

[25] Choi K.M. (2016). Sarcopenia and sarcopenic obesity. Korean J. Intern. Med..

[26] Batsis J.A., Villareal D.T. (2018). Sarcopenic obesity in older adults: Aetiology, epidemiology and treatment strategies. Nat. Rev. Endocrinol..

[27] Li C.W., Yu K., Shyh-Chang N., Jiang Z., Liu T., Ma S., Luo L., Guang L., Liang K., Ma W. (2022). Pathogenesis of sarcopenia and the relationship with fat mass: Descriptive review. J. Cachexia Sarcopenia Muscle.

[28] Hong S.H., Choi K.M. (2020). Sarcopenic Obesity, Insulin Resistance, and Their Implications in Cardiovascular and Metabolic Consequences. Int. J. Mol. Sci..

[29] Ji T., Li Y., Ma L. (2022). Sarcopenic Obesity: An Emerging Public Health Problem. Aging Dis..

[30] Kim T.N., Yang S.J., Yoo H.J., Lim K.I., Kang H.J., Song W., Seo J.A., Kim S.G., Kim N.H., Baik S.H. (2009). Prevalence of sarcopenia and sarcopenic obesity in Korean adults: The Korean sarcopenic obesity study. Int. J. Obes..

[31] Koliaki C., Liatis S., Dalamaga M., Kokkinos A. (2019). Sarcopenic Obesity: Epidemiologic Evidence, Pathophysiology, and Therapeutic Perspectives. Curr. Obes. Rep..

The article "Obesity and Frailty Syndrome in the Elderly: Prospective Study in Primary Care" was retracted in 2024. Reasons: lack of ethics approval or compliance; concerns about the welfare of human subjects.

[32] Choi S., Chon J., Lee S.A., Yoo M.C., Yun Y., Chung S.J., Kim M., Lee E.T., Kyu Choi M., Won C.W. (2022). Central obesity is associated with lower prevalence of sarcopenia in older women, but not in men: A cross-sectional study. BMC Geriatr..

